# Cardiomyocyte Specific Ablation of p53 Is Not Sufficient to Block Doxorubicin Induced Cardiac Fibrosis and Associated Cytoskeletal Changes

**DOI:** 10.1371/journal.pone.0022801

**Published:** 2011-07-28

**Authors:** Tiam Feridooni, Adam Hotchkiss, Sarah Remley-Carr, Yumiko Saga, Kishore B. S. Pasumarthi

**Affiliations:** 1 Department of Pharmacology, Dalhousie University, Halifax, Nova Scotia, Canada; 2 Mammalian Development Laboratory, National Institute of Genetics, Mishima, Shizuoka, Japan; Istituto Dermopatico dell'Immacolata, Italy

## Abstract

Doxorubicin (Dox) is an anthracycline used to effectively treat several forms of cancer. Unfortunately, the use of Dox is limited due to its association with cardiovascular complications which are manifested as acute and chronic cardiotoxicity. The pathophysiological mechanism of Dox induced cardiotoxicity appears to involve increased expression of the tumor suppressor protein p53 in cardiomyocytes, followed by cellular apoptosis. It is not known whether downregulation of p53 expression in cardiomyocytes would result in decreased rates of myocardial fibrosis which occurs in response to cardiomyocyte loss. Further, it is not known whether Dox can induce perivascular necrosis and associated fibrosis in the heart. In this study we measured the effects of acute Dox treatment on myocardial and perivascular apoptosis and fibrosis in a conditional knockout (CKO) mouse model system which harbours inactive p53 alleles specifically in cardiomyocytes. CKO mice treated with a single dose of Dox (20 mg/kg), did not display lower levels of myocardial apoptosis or reactive oxygen and nitrogen species (ROS/RNS) compared to control mice with intact p53 alleles. Interestingly, CKO mice also displayed higher levels of interstitial and perivascular fibrosis compared to controls 3 or 7 days after Dox treatment. Additionally, the decrease in levels of the microtubule protein α-tubulin, which occurs in response to Dox treatment, was not prevented in CKO mice. Overall, these results indicate that selective loss of p53 in cardiomyocytes is not sufficient to prevent Dox induced myocardial ROS/RNS generation, apoptosis, interstitial fibrosis and perivascular fibrosis. Further, these results support a role for p53 independent apoptotic pathways leading to Dox induced myocardial damage and highlight the importance of vascular lesions in Dox induced cardiotoxicity.

## Introduction

Doxorubicin (Dox) is a member of Anthracycline (ANT) family of anticancer drugs. ANTs are frequently administered due to a strong correlation between dose and efficacy [1]. The use of ANTs for cancer treatment can lead to a series of pathophysiological complications such as tumor cell resistance and cellular toxicity. Cardiotoxicity is particularly prevalent in many patients which leads to cardiomyocyte apoptosis, myocardial fibrosis, cardiomyopathy, arrhythmias and congestive heart failure (CHF) [2]. While several distinct mechanisms have been reported as underlying causes of Dox-induced cytotoxicity, it is well established that the tumor suppressor protein p53 plays a key role in Dox-induced apoptosis in cardiomyocytes as well as cancer cells [3].

Dox induces tumor cell apoptosis mainly due to its function as a topoisomerase II (topo-II) inhibitor [4]. The formation of a ternary complex consisting of Dox-DNA-topo II blocks the ligation step of DNA synthesis cycle and causes single and double strand DNA breaks which ultimately leads to cellular apoptosis [5]. In contrast to cancer cells, accumulation of reactive oxygen and nitrogen species (ROS/RNS) and changes in the mitochondrial membrane permeability are the predominant cause of Dox-induced apoptosis in cardiomyocytes and endothelial cells [6]–[8]. Compared to cancer cells, cardiomyocytes are more suceptible to Dox induced free radical damage due to lower levels of catalase [9], an enzyme which serves as a defense mechanism in converting hydrogen peroxide to water and oxygen [10]. It has been proposed that Dox initially increases mitochondrial superoxide and other ROS products via redox cycling followed by generation of NO and other RNS (e.g. peroxynitrite) and subsequently causes an increased expression of NF-κB and inducible nitric oxide synthase (iNOS) [7]. Concerted actions of ROS/RNS have been further implicated in the amplification of oxidative/nitrosactive stress pathways, DNA damage, redox regulation of p53 transcription and posttranslational modifications as well as apoptosis [8]. Some studies have shown that Dox can trigger release of cytochrome c from mitochondria or inhibit electron transport chain and cause apoptosis regardless of DNA damage or p53 levels [11]–[14].

Several cardioprotective approaches have been shown to effectively block Dox induced cardiotoxicity. These include: administration of antioxidants [15], scavengers of peroxynitrite [7], iron chelating agents [16] and glutamate [17], inhibition of endocannabinoids [6], [18], treatment with factors such as erythropoietin [19] or granulocyte stimulating factor [20] and abrogation of p53 activity via global knockdown [21] or chemical inhibition [22] approaches. More recently, Zhu et al. have shown that blocking p53 in a cardiomyocyte restricted manner was sufficient to prevent systolic dysfunction and reduction in cardiac mass induced by acute Dox treatment for seven days [23]. However, these studies did not determine whether short term functional improvement seen in response to p53 abrogation is due to a decreased rate of myocardial fibrosis, a well established risk factor for arrhythmia, cardiomyopathy and CHF [24], [25]. Further, it has not been determined whether Dox administration would lead to perivascular necrosis and associated fibrosis in myocardial tissue from animals with normal or compromised p53 function. Monitoring these aspects is particularly important because Dox treatment is well known to cause a late-onset refractory cardiomyopathy and heart failure [26].

In this study, we have developed a conditional knockout (CKO) mouse model system to facilitate cardiomyocyte specific removal of sequences encoding the p53 gene. To determine whether p53 expression in cardiomyocytes plays any direct role in the onset of cardiac fibrosis in heart tissue, we studied wild type and p53-CKO mice subjected to Dox treatment for various time periods. Reparative myocardial fibrosis reminiscent of myocyte death was present in both wild type and p53-CKO hearts subjected to Dox treatment. We also observed increased incidence of perivascular fibrosis in myocardial sections from Dox treated wild type and p53-CKO mice compared to saline treated mice. Further, we found a significant decrease in the expression levels of α-tubulin, a microtubular protein essential for normal cardiac function, in both wild type and p53-CKO mice 3 days post Dox treatment. Collectively our results suggest that selective loss of p53 in cardiomyocytes is not sufficient to block myocardial fibrosis and loss of microtubule proteins in acute phase of Dox treatment. These results underscore the importance of p53 independent pathways as well as vascular lesions in Dox induced cardiotoxicity.

## Materials and Methods

### Ethics Statement

All animal procedures were performed according to the Canadian Council on Animal Care guidelines and were approved by the Dalhousie University Committee on Laboratory Animal Care (Protocol#10-008; 09-038).

### Generation and Genotyping of Mice

Cardiomyocyte specific deletion of p53 was accomplished by Cre-lox based technology. Generation of mice with Cre recombinase inserted into the coding sequence of Mesp1 was previously described [27]. Mesp1 is expressed in early mesoderm at the onset of gastrulation, including heart precursor cells. Only Mesp1-Cre heterozygous mice (MC^+/−^) were used in this study as the homozygous Cre mice (MC^+/+^) were embryonic lethal [27]. Similarly, generation of mice with loxP sites inserted into introns 1 and 10 of the p53 gene (p53 floxed allele or p53^F2-10^, Figure 1A) was previously described [28]. Both strains of mice were maintained in C57BL6/J (BL6) background. For control comparisons, BL6 and CD1 mice were purchased from Jackson (Maine, MA) and Chrales River Laboratories (Wilmington) respectively. Efficient Cre mediated removal of the p53 coding sequence between loxP sites was accomplished by crossing floxed p53^F2-10^ mice (heterozygous designated p53^F/+^ and homozygous designated p53^F/F^) with mice expressing Mesp1-Cre (designated MC^+^). To confirm the genotype of offsprings, genomic DNA was extracted from ear punch biopsies and a polymerase chain reaction (PCR) amplification assay was performed using RedExtract amplification kit (Sigma) and appropriate primer sets for MC and p53 transgenes (Fig. 1A and B, see Table 1 for sequences). To confirm the deletion of exons 2–10 corresponding to p53 allele (p53^ΔF2-10^, Fig. 1A), genomic DNA was extracted from heart tissue and PCR was performed using primer pairs 1FA and 10RA (Fig. 1C and Table 1). PCR conditions for MC transgene amplification were *95°C 30 sec, 60°C 30 sec, 72°C 30 sec for 30 cycles*. Similarly, PCR conditions for p53 alleles were *94°C 30 sec, 68°C 1 min, 72°C 2 min for 30 cycles*.

**Figure 1:** Generation and characterization of p53 conditional knockout mice. (**A**) Schematic representation of transgenic alleles corresponding to MesP1-Cre (MC), floxed p53 (p53^F2-10^) and conditional p53 deletion (p53^ΔF2-10^) mice. Positions of exons and loxP sites are indicated by numbered black boxes and arrowheads respectively. Positions of primer pairs used for genotyping are indicated by arrows. (**B**) MC positive (+) and negative (−) mice were identified by PCR amplification of ear punch genomic DNA using NeoAL and GR1 primers. Mice homozygous (F/F) or heterozygous (F/+) for floxed p53 alleles were identified using 10FM and 10RM primers. Wt: wild type; H2O: no template control for PCR. (**C**) Excision of exons 2–10 of p53 gene in double transgenic hearts (MC^+^ and p53^F/F^ or ^F/+^) was confirmed by PCR amplification of cardiac genomic DNA using 1FA and 10RA primers. Note the absence of PCR amplification product with 1FA/10RA primers in MC^−^ p53^F/F^ mice. Excision of p53 exons does not occur in MesP1 negative non-cardiacmyocytes. As a result, primers specific for intron 10 (10FA/10RA) and intron 1 (1FA/1RA) can also amplify PCR products from cardiac genomic DNA.

**Table 1:** Primers used for genotyping analysis.

Gene	Primer pairs (5′ to 3′)	Amplicon size (bp)
MesP1-Cre	Neo AL: GAAAGAACCAGCTGGGGCTCGAG	1080
	GR1: ATATGCCAAGTCATTGAGGTGAGCTTTC	
p53 Floxed allele (intron 10)	10FM: AAGCTGAAGACAGAAAAGGGGAGGG	585 (floxed allele)
	10RM: AAGCTAAGGGGTATGAGGGACAAGG	432 (wild type)
p53 Floxed allele (intron 10)	10FA: GTAAGTGGCCTGGGGCAGCG	722 (floxed allele)
	10RA: GGGGAGGGATGAAGTGATGGGAGC	569 (wild type)
p53 Floxed allele (intron 1)	1FA: GCGACTGACTGTGCCCTCCGT	450 (floxed allele)
	1RA: GGAACCATCGCTTTCGCACCTTGG	368 (wild type)
p53 Deletion allele (p53^ΔF2-10^)	1FA: GCGACTGACTGTGCCCTCCGT	603
	10RA: GGGGAGGGATGAAGTGATGGGAGC	

### Doxorubicin Injections and Sample preparation

MC^+^p53^F/F^ and MC^+^p53^F/+^ male mice aged 11–15 weeks were injected intraperitoneally with a single dose of either Doxorubicin Hydrochloride (20 mg/kg, Mayne Pharma, Montreal, QC) or saline. Age and sex matched control BL6 mice which were negative for either the MC transgene or p53 floxed allele were also processed using the same injection protocol. Mice were sacrificed by cervical dislocation after 3 or 7 days post Dox injection and heart tissues were subsequently collected, weighed and divided into three parts. The top third of each heart was stored at −80°C and subsequently used for p53 western blot analysis. The bottom two thirds were placed in 30% sucrose solution overnight at 4° for cryoprotection, subsequently embedded in tissue freezing medium (Tissue-tek, O.C.T., Sakura Finetek, Japan), frozen at −80°C and processed for histological analysis. Thin tissue sections (10 µm) were generated using a Leica CM 3050 S Cyrostat. Heart weight to body weight ratios were calculated to examine whether the genomic modification had any significant impact on the physiology of the mice. Each treatment group consisted of three to five mice. For a comparison of myocardial fibrotic lesions induced by Dox with those induced by excessive catecholamines, cardiac hypertrophy was induced in 11–15 week old male CD1 mice by implanting mini-osmotic pumps filled with sterile saline containing isoproterenol as described in our earlier study [29].

### Immunofluorescence staining of Myocardial Sections

To study the effect of Dox treatment on p53 expression, thin cryosections were generated as described earlier [30]. Sections were fixed in methanol for 15 minutes at 4°C and blocked with 10% goat serum and 1% bovine serum albumin (BSA) in PBS for 60 minutes. Parallel sections were incubated with rabbit polyclonal antibodies directed against p53 (SC-6243; Santa Cruz Biotechnology, Santa Cruz, CA, USA) or Von Willebrand Factor (VWF, SC-14014; Santa Cruz Biotechnology, Santa Cruz, CA, USA). Sections were subsequently incubated with goat anti-rabbit secondary antibodies conjugated to Alexa Fluor 555 (Invitrogen, Carlsbad, CA, USA) for those probed for p53 expression or Alexa Fluor 488 (Invitrogen, Carlsbad, CA, USA) for those probed for VWF protein. Nuclei were stained with 10 µg/ml of Hoechst 33342 for 5 minutes. Samples were mounted in 1% propyl gallate solution and examined using a Leica DM2500 fluorescence microscope (Leica Microsystem). Images were captured using a Leica DFC 500 digital acquisition system.

### Polyacrylamide Gel Electrophoresis (PAGE) and Western Blot Analysis

Mouse hearts were homogenized in tumor lysis buffer [1% NP40, 5 mM EDTA, 50 mM Tris-HCl pH 8.0, phenylmethylsulphonyl fluoride (PMSF; 10 µg/ml) and aprotinin (10 µg/ml)] as described earlier [31]. Lysates were sonicated and centrifuged at 13,500 rpm for 15 minutes at 4°C. Supernatants were collected and protein concentrations were estimated by the Bradford assay (Pierce). 40 µg of protein was denatured in Laemmli buffer and separated in denaturing conditions on a 12.5% SDS-PAGE gel and transferred onto a nitrocellulose membrane. Blots were routinely stained with 0.1% Naphthol blue black (Sigma-Aldrich) to determine the amount of protein loading. Membranes were blocked (5% milk, 3% BSA, 0.1% Tween in PBS), and incubated with antibodies specific for p53 (SC-6243), CBF-A (SC-13045) and α-tubulin (SC-8035) followed by incubation with anti-rabbit or anti-mouse antibodies conjugated to horse radish peroxidase. Signals were visualized using the ECL method (GE Healthcare). In some cases, imaging films were scanned and analyzed by NIH ImageJ software. The linear range of a density curve was selected for calculations. The levels of α-tubulin were normalized to those of CBF-A for each sample in order to correct for any variations in protein loads. Adjusted values were further normalized to the protein levels in the control saline treated samples. The densitometry data are presented as relative changes from control levels ± SEM.

### Terminal deoxynucleotidyl transferase-mediated dUTP Nick End Labelling (TUNEL) and Active Caspase 3 (Casp3) Staining

The TUNEL assay was performed for detection of apoptosis in myocardial sections using TMR Red *In Situ* cell death detection kit according to manufacturer's instructions (Roche Applied Science, Mannheim, Germany). Slides were fixed in 4% paraformaldehyde for 1 hour at room temperature, processed for TUNEL assay, then washed with PBS and labelled with Hoechst 33258 (10 µg/µl) at room temperature for 3 minutes. Subsequently, slides were rinsed with PBS and mounted with propyl gallate solution. Apoptotic cells were detected using a Lecia DM2500 microscope with appropriate filters. Negative control consisted of the labelling solution without the enzyme solution.

For active Caspase 3 (Casp3) staining, cryosections were hydrated in PBS and fixed in formalin for 15 min. Sections were subsequently quenched in 0.3% hydrogen peroxide for 30 min, blocked for 5 hours and incubated with anti-active Casp3 antibody (G7481, Promega, Madison) overnight at 4°C followed by secondary antibody detection reagents from Vectastain ABC system (Vector Labs) according to the instructions provided by the supplier. Signal was visualized using the diaminobenzidine (DAB) solution (1 DAB tablet (Sigma), 0.375 g Nickel Ammonium Sulfate and 1.5 ml of 3% hydrogen peroxide dissolved in 62.5 ml of TBS, pH 8). Slides were immersed in DAB solution for 10 min, dehydrated in graded ethanol (70%, 95% and 100%), xylene and mounted using cytoseal-60 (Richard-Allan Scientific). All Casp3 staining steps were performed at room temperature unless otherwise specified.

### Assessment of Superoxide and 3-Nitrotyrosine (3-NT) Levels in Myocardial Sections

Unfixed cryosections were hydrated in PBS, incubated with 5 µM dihydroethidium (DHE, Invitrogen) at 37°C for 30 min, rinsed with PBS and mounted using propyl gallate solution. DHE fluorescence was imaged using a Zeiss LSM 510 Meta confocal microscope as recommended in previous studies [32]. For detection of 3-NT, cryosections were fixed and immunostained with 3-NT antibodies (#sc-55256, Santa Cruz, CA) using Vectastain ABC system similar to that described for Casp3 staining procedure.

### Quantification of Fibrosis

To determine the extent of fibrosis due to Dox treatment, cryosections were processed for Picro Sirius Red and Fast Green staining as described earlier [29]. Slides were fixed in Bouins solution at 55°C for 1 hour, washed with water, stained with 0.1% Fast Green (Sigma) at room temperature for 10 minutes, washed with 0.1% acetic acid for two minutes, and stained with 0.1% Pico Sirius Red for 30 minutes (Sigma-Direct red 80 in saturated aqueous picric acid). The slides were dehydrated in an ascending grade of 70, 95, and 100% ethanol for approximately 2 minutes per wash, cleared in xylene solution for 2 minutes and mounted in cytoseal-60. Quantification of cardiac fibrosis was performed via Colour-Subtractive Computer-Assisted Image Analysis (CS-CAIA) as described previously [29]. Areas occupied by green pixels (representing healthy cardiac tissue) and areas occupied with red pixels (representing fibrotic tissue) from photomicrographs were assessed by an image processing software developed by Reindeer Graphics (Asheville, NC, USA). Percent fibrosis was calculated based on the area occupied by red pixels divided by the sum of area occupied by red and green pixels multiplied by one hundred. Each treatment group consisted of three to five mice, of which ten sections per heart were sampled for fibrosis quantification.

### Statistical Analysis

Data are presented as the mean ± SEM. Multiple group comparisons for heart weight body weight ratios, active caspase levels, fibrosis assessment, α-tubulin and CBF-A levels were analyzed by ANOVA with Tukey's multiple comparison tests using Graphpad Prism 4 (GraphPad software, San Diego, CA). Significance was assumed at *P*<0.05.

## Results

### Conditional excision of p53 exons 2–10 in adult mouse cardiomyocytes

The aim of this study was to determine the role of p53 expression in cardiomyocytes and vascular cells in the context of Dox-induced cardiotoxicity. To this end, we crossed mice expressing Cre recombinase exclusively in cardiomyocytes (MC^+^) with mice harboring floxed p53^F2-10^ alleles and generated cardiomyocyte specific p53 CKO mice (Fig. 1A). The MC^+^ offsprings could be readily identified by amplification of a 1080 bp fragment from the ear punch genomic DNA using NeoAL and GR1 primers (Fig. 1B and Table 1). PCR amplification of ear punch genomic DNA using intron 10 specific primers of p53 (10FM/10RM) yielded 585 bp and or 432 bp products. Amplification of both fragments confirmed the identity of mice as heterozygous for floxed p53^F2-10^ allele (p53^F/+^). In contrast, mice homozygous for floxed (p53^F/F^) or wild type p53 alleles were identified by exclusive amplification of 585 bp or 432 bp bands respectively (Fig. 1B). Similarly, another intron 10 specific primer pair (10FA/10RA) and intron 1 specific primer pair (1FA/1RA) were also used to identify p53^F/+^, p53^F/F^ and wild type genotypes (Table 1). Using this Cre-lox approach, sequences corresponding to exons 2–10 of p53 allele are expected to remain intact in non-cardiac tissue. Accordingly, all p53 primer pairs could efficiently amplify appropriate size fragments from ear punch DNA of wild type or transgenic mice.

In contrast to ear punch biopsies, expression of Cre recombinase in MC^+^ p53^F/+^ or MC^+^p53^F/F^ double transgenic hearts is expected to facilitate excision of exons 2–10 of p53 allele exclusively in cardiomyocytes. This is due to the fact that Mesp1 transcription factor is expressed in early cardiomyocyte precursor cells but not in vascular smooth muscle cells (VSMC), endothelial cells (EC) and any other ecto- or endoderm derived cells. In agreement with this notion, amplification of the genomic DNA isolated from double transgenic heart tissue (MC^+^p53^F/+^ or MC^+^p53^F/F^) using 1FA and 10RA primers which span introns 1–10 of p53 gene resulted in a 603 bp product (Fig. 1C). However, 1FA/10RA primer pair failed to amplify any product from cardiac genomic DNA in the absence of Cre expression (Fig. 1C). As expected, primers specific for both intron 10 (10FA/10RA) and intron 1 (1FA/1RA) were also able to amplify appropriate size PCR fragments from cardiac genomic DNA of the double transgenic hearts accounting for intact p53 floxed alleles present in non-cardiomyocyte cell types (Fig. 1C). There was no evidence of altered cardiac growth either in MC^+^p53^F/+^ or MC^+^p53^F/F^ compared to wild type BL6 mice (11–15 week old mice were examined). Similarly, histological analyses did not reveal any overt changes such as hypertrophy or fibrosis as a result of genetic modifications in double transgenic hearts (data not shown). Furthermore, the cardiac specific p53 CKO mice did not develop tumors such as those frequently observed in conventional p53 knockouts [28].

### Assessment of p53 expression profiles and apoptosis levels in wild type and p53 CKO hearts treated with or without Doxorubicin

Consistent with previous studies [23], [33], we observed very low levels of p53 expression in untreated and saline treated wild type or CKO mouse hearts using immune histology and western blot analysis methods (Fig. 2A and D). In case of wild type hearts treated with Dox, p53 expression was readily detectable in both nuclear and cytoplasmic compartments of cardiomyocytes as well as vascular cells at 3 and 6 hrs post drug treatment (Fig. 2B and C). In contrast to wild type hearts, p53 immunostaining was observed only in vascular cells but not in cardiomyocytes of MC^+^p53^F/F^ CKO mice (Fig. 3A). Parallel sections processed for VWF staining confirmed that endothelial cells account in part for the increased levels of p53 observed in myocardial blood vessels (Fig. 3B). The VWF staining intensity was much higher in Dox treated hearts compared to untreated or saline treated hearts. Further, VWF immunostaining revealed high concentrations of protein in subendothelial matrix (Fig. 3B). Based upon western blotting studies, p53 protein levels decreased in both wild type and CKO mice after 7 days of Dox treatment and were comparable to those observed in control hearts (Fig. 2D).

**Figure 2:** Expression of p53 in the heart after Dox treatment. (**A**) Very low levels of p53 immunostaining were observed in the control untreated heart. (**B and C**) Increased expression of p53 was evident in cytoplasmic and nuclear compartments of cardiomyocytes in hearts treated with Dox for 3 or 6 hrs. Bar, 20 µm (A–C). (**D**) Western blot analysis of p53 protein levels in wild type (WT) and p53 conditional knockout (MC^+^ and p53^F/F^ or ^F/+^) hearts treated with saline (S) or Dox (D) for 3 days (3 d) or 7 days (7 d). A 25 kD band from Naphthol Blue Black stained blots was used as a loading control (LC) for protein loading.

**Figure 3:** Expression of p53 and TUNEL staining in vascular cells after 3 day Dox treatment in MC^+^ p53^F/F^ conditional knockout hearts. Cardiac sections were processed for p53 (A), VWF (B) and nuclear (C) staining. Bar, 50 µm (A–C). (**D**) Examples of TUNEL positive vascular cells in MC^+^ p53^F/+^ hearts after 3 day Dox treatment. (**E**) Examples of TUNEL positive cardiomyocytes in MC^+^ p53^F/F^ hearts. Bars, 50 µm, D and E.

The cardiotoxic effects of Dox are partly attributed to induction of apoptotic pathways involving p53 [13], [21], [22]. A hallmark of apoptosis is activation of endonucleases that are responsible cleavage of chromosomal DNA at internucleosomal linker regions. To determine the levels of apoptosis in Dox treated hearts, a TUNEL assay was used. This assay is based on the detection of single or double stranded DNA breaks by *in situ* terminal deoxynucleotidyl transferase labelling with a fluorochrome which allows apoptotic nuclei to be readily distinguished from healthy nuclei. While control sections showed very low levels of TUNEL activity, considerably larger number of TUNEL positive nuclei were detected in Dox treated wild type hearts from 3 and 7 day time points (∼100–200 per square millimetre). A similar level of apoptosis was also detected in sections from Dox treated p53 CKO mice. Interestingly, TUNEL positive nuclei were found in cardiomyocytes, interstitial and vascular regions after Dox treatment independent of p53 status in all experimental groups (Fig. 3D and E).

Immunostaining of heart sections with antibodies specific for active caspase 3 (Casp3^+^) indicated that both cardiomyocytes and vascular cells can undergo caspase dependent apoptosis in Dox treated wild type and p53 CKO mice (Fig. 4). Compared to the control value, number of Casp3^+^ cardiomyocytes per mm^2^ was significantly higher in Dox treated wild type or p53 CKO hearts at 3 day time point (∼2 or ∼5 fold respectively, Fig. 4B). Further, Casp3^+^ numbers in Dox treated MC^+^p53^F/F^ hearts were significantly higher (∼2 fold) than those observed in Dox treated wild type hearts (Fig. 4B).

**Figure 4:** Caspase dependent apoptosis after 3 day Dox treatment in MC^+^ p53^F/F^ conditional knockout hearts. (**A**) Examples of cardiomyocytes positive for active caspase 3 in myocardial sections, Bar, 20 µm, (**B**) Quantification of caspase 3 positive cardiomyocytes per mm^2^ in saline (S) or Dox (D) treated wild type (WT) or p53 CKO hearts. N = 3 mice per group, *P<0.05 compared to WT(S), #*P*<0.005 compared to WT(S) or WT(D), ANOVA, Tukey's multiple comparisons test.

### Assessment of ROS and 3-NT levels in wild type and p53 CKO hearts treated with or without Doxorubicin

Given the increased levels of myocardial apoptosis in p53 CKO hearts, we subsequently examined the levels of ROS by DHE staining (Fig. 5). Membrane permeable DHE has been widely used as a detection probe for superoxide and other ROS, since its oxidation product ethidium can be readily detected by fluorescence microscopy [7], [32]. DHE fluorescence signal was observed mainly in endothelial and smooth muscle cells of wild type saline treated hearts at 3 day time point (Fig. 5A). In contrast, DHE staining was observed at a higher frequency in vascular cells as well as cardiomyocytes in the hearts of Dox treated wild type or p53 CKO mice (Fig. 5B, C). To assess the nitrosactive stress caused by peroxinitrite pathway, sections were also examined using 3-NT immunohistochemical staining. Compared to a smaller number of 3-NT positive cells in saline treated hearts, a higher frequency of 3-NT positive cardiomyocytes and vascular cells was observed in Dox treated wild type and p53 CKO hearts at 3 day time point (Fig. 5D–F). These findings collectively suggest that Dox treatment can increase ROS and RNS generation and trigger caspase dependent apoptosis independent of p53 status in cardiomyocytes.

**Figure 5:** Dox treatment induces ROS and 3-nitrotyrosine generation independent of p53 gene status in the heart. (A–C) Detection of superoxide/ROS after 3 day Dox treatment in frozen sections of wild type or p53 CKO hearts using dihydroethidium (DHE) staining. (**A, B**) DHE positive endothelial or smooth muscle cells in saline (S) or Dox (D) treated wild type (WT) hearts are indicated by arrows. (**C**) Examples of DHE positive cardiomyocytes are indicated by arrowheads. Bar, 50 µm, A–C. (**D–F**) Immunostaining of 3-nitrotyrosine (3-NT) in sections derived from saline (S) or Dox (D) treated WT (D, E) and p53 CKO (F) hearts at 3 day time point. Note the increase in 3-NT staining in cardiomyocytes after DOX treatment in both WT and p53 CKO hearts. Bar, 50 µm, D–F.

### Assessment of cardiac fibrosis levels in wild type and p53 CKO hearts treated with or without Doxorubicin

Given the higher incidence of apoptosis and free radical generation in Dox treated p53 CKO hearts, we further examined whether ablation of p53 in cardiomyocytes is sufficient to prevent Dox induced cardiac fibrosis. Since adult myocardium lacks intrinsic regenerative capacity, dead cardiomyocytes are replaced by scar tissue, a process often referred to as reparative fibrosis [34], [35]. Picro Sirius red (PS) and fast green (FG) stains can be used to distinguish fibrotic regions from healthy myocardium [29]. Histological sections from wild type and p53 CKO mice were stained with PSFG stain and examined under a microscope to identify fibrotic lesions (Fig. 6A–D). Histologically, Dox treatment induced both reparative and perivascular types of fibrosis in wild type hearts compared to background level of fibrosis in saline treated hearts (Fig. 6A,B). In agreement with apoptotic cells found, both reparative as well as perivascular fibrosis were also observed in the hearts of Dox treated p53 CKO mice (Fig. 6C, D). In the presence of sustained catecholamine mediated cardiac injury, reparative fibrosis was shown to switch into reactive fibrosis, a process characterized by increased deposition of collagen and extracellular matrix (ECM) in interstitial areas remote to the site of injury [29]. Typically, the spread of Dox induced fibrotic lesions was ∼2.5 times smaller than that of Iso induced lesions (Mean lesion lengths ± SEM: Dox = 303±15 µm vs. Iso = 815±33 µm, Fig. 6E). Although there was a slight decrease in heart weight to body weight ratio (HW/BW) of Dox treated wild type mice compared to saline treated group, Dox treatment did not have any effect on HW/BW ratios of p53 CKO mice (Fig. 6F).

**Figure 6:** Dox treatment induces myocardial fibrosis independent of p53 gene status in the heart. (**A–D**) Representative photomicrographs of PSFG stained cardiac sections from wild type or p53 CKO hearts treated with saline (A) or Dox (B–D) at 7 day time point. Both reparative (C) and perivascular (D) types of fibrosis were evident in Dox treated MC^+^ p53^F/F^ conditional knockout hearts. Bar, 100 µm A–D. (**E**) Quantification of the spread of cardiac fibrosis lesions in Dox and Isoporterenol (ISO) treated hearts at 7 day time point. LL: lesion length, LW: lesion width. ISO induced LL was significantly greater (∼2.5 fold) compared to Dox induced LL (n = 3–5 mice per group, *P<0.005 compared with other groups. ANOVA, Tukey's multiple comparison test). (**F**) No significant difference is observed between groups in heart weight and body weight ratios of mice used in these studies at 7 day time point.

To quantify the fibrotic areas in tissue sections, CS-CAIA software was used as previously described [29]. The fibrotic area from each section was then expressed as percent fibrosis. The control group for three day time point showed a basal fibrosis of 2% (Fig. 7A). Compared to the control value, the percent fibrosis was significantly higher in Dox treated wild type or p53 CKO hearts at 3 day time point (Fig. 7A). Interestingly, fibrosis levels in Dox treated MC^+^p53^F/F^ hearts were significantly higher (∼2 fold) than those observed in Dox treated wild type hearts at 3 day time point (Fig. 7A). A similar trend in fibrosis levels was also observed at 7 day time point. Compared to the control fibrosis levels, Dox treatment led to significantly higher levels of fibrosis in all experimental groups irrespective of p53 status at 7 day time point (Fig. 7B). Further, fibrosis levels decreased by 25–50% in Dox treated hearts at 7 day time point compared to 3 day time point (Fig. 7A and B). Thus, our results suggest that conditional ablation of p53 in cardiomyocytes does not offer protection against cardiac fibrosis induced by Dox.

**Figure 7:** Quantification of cardiac fibrosis in tissue sections after 3 or 7 days of Dox treatment. Percent fibrosis values in PSFG-stained heart sections were calculated using Image processing Tool Kit software and image analysis was performed on a minimum of ten slides per animal for each treatment group (n = 3–5 mice per group). Dox (D) treatment significantly increased cardiac fibrosis in wild type (WT) and p53 CKO hearts compared to saline (S) treated hearts after 3 day (A) or 7 day (B) treatment periods. 3 day Dox time point: *P<0.05 compared to WT(S), **P<0.05 compared to WT(D), ANOVA, Tukey's multiple comparisons test; 7 day Dox time point: #*P*<0.05 compared to WT(S), ANOVA, Tukey's multiple comparison test.

### Assessment of α-tubulin protein levels in wild type and p53 CKO hearts treated with or without Doxorubicin

Previous studies have shown that administration of a normal therapeutic dose of Dox can alter the expression profiles of some cytoskeletal and ECM proteins in the rat heart [36]. Using cultured chick cardiomyocytes, it was shown that Dox treatment could lead to damage of microtubule structures and impairment of microtubule assembly [37]. Given the previous reports on improved cardiac function after Dox treatment in p53 global knockout mice, we have examined whether ablation of p53 in cardiomyocytes is sufficient to prevent microtubule changes reported earlier. To quantify levels of detergent soluble α-tubulin protein, cytosolic fractions were prepared from saline or Dox treated control and p53 CKO mouse hearts at 3 or 7 day time points, western blotting and densitometry were performed as described in methods section. We normalized α-tubulin levels to those of CBF-A as we did not find any significant changes in CBF-A levels with or without drug treatment in control and p53 CKO hearts (data not shown). Compared to the control value, normalized α-tubulin levels were significantly lower (∼2–2.5 fold) in Dox treated wild type or p53 CKO hearts at 3 day time point (Fig. 8A). However, there was no significant difference in α-tubulin levels between Dox treated wild type, MC^+^p53^F/F^ or MC^+^p53^F/+^ hearts (Fig. 8A). Seven days after Dox treatment, α-tubulin levels in all Dox treated groups returned back to those seen in control hearts (Fig. 8B). Thus, our results suggest that conditional ablation of p53 in cardiomyocytes is not adequate to prevent microtubule changes associated with Dox treatment.

**Figure 8:** Quantification of α-tubulin levels in the hearts of Dox treated and control mice. Ventricular lysates were analyzed 3 days (A) and 7 days (B) after saline (S) or Dox (D) treatment. The levels of α-tubulin were normalized to those of CBF-A for each sample and ratios were expressed as fold changes relative to WT(S) (n = 3 hearts per group). (**A**) Following a 3 day treatment period, α-tubulin/CBF-A ratios were significantly lower in Dox treated hearts (both wild type (WT) and p53 CKO) compared to those ratios in saline treated hearts. *P<0.05 compared to WT(S), ANOVA, Tukey's multiple comparison test. (**B**) Following a 7 day treatment period, α-tubulin/CBF-A ratios were not significantly different between Dox (D) or saline (S) treated hearts.

## Discussion

Dox undergoes a redox reaction in cardiac mitochondria, where it is reduced by NADH dehydrogenase to form a semiquinone compound which is oxidized back to the original structure by transferring an electron to the molecular oxygen. This process generates ROS including superoxide, hydrogen peroxide and hydroxyl radicals (Fig. 9, [3], [38]). Excessive superoxide can react with nitric oxide to generate RNS such as peroxynitrite [3], [7], [38]. Iron has been shown to promote ROS formation in Dox treated cells [38]. Further, a variety of factors are known to amplify ROS/RNS mediated oxidative/nitrosactive stress which leads to strand breaks in DNA, activation of poly ADP ribose polymerase, DNA damage, upregulation of redox sensitive transcription factors such as p53 and NF-κB, changes in mitochondrial permeability, apoptosis and ultimately cardiotoxicity (Fig. 9, [7], [8], [39]). Overexpression of manganese superoxide dismutase or treatment with peroxinitrite scavengers have been shown to decrease ROS/RNS generation and mitochondrial injury [7], [40]. While the majority of studies highlight the importance of ROS in cardiotoxicity, some studies have proposed that RNS is the major cause of cardiotoxicity [7]. Although several experimental strategies have been suggested for prevention of Dox-induced cardiotoxicity [3], [38], numerous preclinical/clinical studies have led to negative or mixed outcomes suggesting a role for alternate mechanisms other than the conventional ROS and iron based hypotheses [38]. Understanding different cytotoxic mechanisms of Dox is critical to prevent cardiotoxic effects when using this drug for anticancer therapies. Recent studies have indicated that abating the function or deleting p53 in myocardium may decrease Dox-induced cardiotoxicity and improve left ventricular ejection fraction [21], [23]. However, none of these studies directly compared levels of cardiac fibrosis or incidence of myocardial vascular lesions in response to drug treatment in animals with intact or deleted p53 gene. This is particularly important since Dox concentrations were shown to be significantly higher in perivascular areas compared to hypoxic regions in solid tumors [41]. A similar distribution pattern of Dox in heart tissue may lead to an increased incidence of perivascular lesions limiting oxygen supply to adjacent myocytes. In this study, we found that cardiomyocyte specific disruption of p53 gene does not reduce levels of free radical generation, apoptosis and myocardial fibrosis or vascular lesions.

**Figure 9:** Schematic representation of mechanisms underlying DOX-induced cardiotoxicity. Redox recycling of DOX in mitochondria results in increased levels of superoxide and subsequent generation of other types of reactive oxygen and nitrogen species (ROS/RNS). Increased levels of ROS results in activation of NF-κB leading to expression of iNOS and thus increased NO expression. Peroxynitrite formation in both mitochondria and cytosol leads to activation of stress signaling pathways such as MAPKs. Build-up of ROS results in expression of phosphorylated p53 which in turn activates the BAX gene. BAX is involved in cytochrome c release from the mitochondria which leads to activation of Caspase 3/7 pathway eventually causing apoptosis. In the absence of p53, negative feedback regulation of ROS and iNOS is lost, which leads to upregulation of reactive oxygen/nitrosactive stress. BAX gene is transcriptionally active in p53 null cells. Excessive ROS/RNS can cause translocation of BAX to mitochondria eventually leading to apoptosis. Further, p53 plays an essential role in mitochondrial DNA repair, and in the absence of p53 this process is hindered. **Note:** * or red arrows denote potential steps effected/involved in Dox induced cell death in p53 CKO cardiomyocytes. O_2_^.−^: superoxide; ONOO^−^: peroxynitrite; ^.^OH: hydroxyl radical; H_2_O_2_: hydrogen peroxide; MnSOD: manganese superoxide dismutase; MAPK: mitogen activated protein kinase; MAP4: microtubule associated protein 4; iNOS: inducible nitric oxide synthase; Ref1: redox effector factor 1; TF: transcription factor.

Expression of p53 appears to be tightly regulated in the myocardium since very low levels of transcripts or protein were found in normal and hypertrophic murine adult hearts [23], [33]. In contrast, the percentage of immunoreactive p53 nuclei was shown to significantly increase (∼4 fold) in myocardial biopsies obtained from end-stage heart failure patients compared to those from normal patients which suggests a role for this cell cycle regulatory protein in cardiomyocyte death [42]. It is generally accepted that changes in p53 protein levels as well as its phosphorylation status play a crucial role during Dox induced cardiotoxicity [3], [22]. However, there are conflicting reports with regards to timing and cardiac expression levels of p53 after Dox treatment. For instance, several studies reported that peak levels of p53 expression ranged from 3–8 hrs and its expression lasted for 24 hrs to 7 days post Dox treatment [13], [22], [23], [43]. In this study, we found that p53 expression was readily detectable in both nuclear and cytoplasmic compartments of cardiomyocytes as early as 3 hrs post Dox treatment of wild type but not p53 CKO mice (Fig. 2). Compared to previous reports, we were unable to detect any significant differences in p53 expression levels between control and Dox treated hearts during 24 hrs to 7 days after treatment (Fig. 2D). Such variations in p53 expression can be attributed to differences in mouse strains and or dosing regimens used in these studies.

Dox treatment also increased p53 levels in vascular endothelial cells in both wild type and CKO mouse hearts (Fig. 3A). Consistent with a proapoptosis role for p53, we observed an increased incidence of Casp3^+^ and TUNEL positive vascular cells with a concomitant increase in perivascular fibrosis in both wild type and p53 CKO hearts (Figs. 3D and 4). We have also observed a similar pattern of Dox induced perivascular fibrosis in p53 CKO generated by an independent cardiomyocyte specific Cre expression line, Nkx2.5-Cre (data not shown). These observations are directly in agreement with previous *in vitro* studies which documented p53 dependent apoptosis in Dox treated human umbilical vein endothelial cell cultures [44], [45]. Accumulation of VWF in subendothelial matrix in our study is consistent with Dox induced vascular damage since elevated levels of VWF were reported during the course of acute coronary syndrome or thromboembolyic cardiovascular events [46]. Collectively, our data shows that myocardial vascular lesions also play a critical role in Dox induced cardiotoxicity.

In addition to vascular lesions, increased levels of apoptosis were also observed in cadiomyocytes from Dox treated WT and CKO hearts. Given the established role of p53 in Dox induced cardiomyocyte death, it is somewhat unexpected to see an increase in the number of TUNEL and Casp3 positive cardiomyocytes in p53 CKO mice. However, this result may be explained in several ways. First, increased incidence of perivascular lesions may limit supply of oxygen and nutrients and trigger ischemic cell death in adjacent cardiomyocytes. Second, recently described but not well characterized p53 independent cell death pathways [47], [48] may also play a role in Dox induced cardiomyocyte death in p53 CKO mice. Dox was shown to induce cell death in p53 null Saos-2 cells via a ROS and Casp3 dependent pathway [49]. Although our data shows increased activation of Casp3 in p53 CKO cardiomyocytes, a role for Dox induced calpain dependent and Casp3 independent cell death pathway cannot be completely ruled out [50]. Third, contrary to the majority of previous reports, loss of p53 in cardiomyocytes can compromise cell survival following Dox treatment. Indeed, a global loss of p53 was shown to increase cardiomyocyte mitochondrial vulnerability to damage following Dox treatment [13]. Similarly, loss of p53 was associated with increased production of ROS and iNOS [51], [52] and increased sensitization to NO induced apoptosis [51] in noncardiac cell types of p53 knockout mice. Further, loss or downregulation of p53 was shown to cause excessive oxidative damage of DNA [53]. Taken together, these studies suggests that p53 regulates a negative feedback loop which controls the production of cellular ROS and RNS [51]–[53]. Based on these earlier studies, absence of p53 in CKO cardiomyocytes is expected to increase ROS, RNS, DNA damage and cell death when subjected to Dox treatment. Consistent with this notion, our data shows significant increases in ROS/RNS, TUNEL and active Casp3 levels in p53 CKO cardiomyocytes after Dox treatment. Fourth, ROS and RNS may directly release cytochrome c from mitochondria [11]–[13] or increase the translocation of Bax to mitochondria [54] thus inducing apoptosis independent of p53. Significant differences in the levels of ROS/RNS, active Casp3 and fibrosis in Dox treated p53 CKO hearts compared to Dox treated wild type hearts at 3 day time point clearly supports a protective role for p53 in cardiomyocytes during Dox induced cardiotoxicity as described in an earlier report [13].

Loss of collagen matrix and cardiac remodelling have been shown to occur for several weeks after a single Dox injection [55], [56]. Even after the drug is removed from the circulation and cardiac tissue, mitochondrial dysfunction, cell death and remodelling changes continue to occur due to an amplification of oxidative and nitrosactive stress pathways [7]. While there is scant information on the development of myocardial fibrosis in an acute setting similar to that described in this study, Dox induced cardiac fibrosis has been reported in several long term studies [57], [58]. One of these long term studies showed absence of cardiac fibrosis in wild type mice 5 days after Dox administration [58]. Such differences in cardiac fibrosis can be attributed to differences in mouse strains, starting age for Dox treatment, time points, staining techniques and dosing regimens used in these studies. Further, upregulation of different matrix metalloproteases (MMPs 1, 2 and 9) has been reported in both short and long term settings of Dox treatment in animal and cell culture models [7], [59]–[61]. In the absence of sufficient quantities of tissue inhibitors of metalloproteases (TIMPs), activated MMPs can digest collagen matrix and ECM and trigger reparative fibrosis in Dox induced or dilated cardiomyopathy [59], [61], [62]. Although we have not measured MMP levels in our study, differences in the time course of MMP activation may also account for the early onset of fibrosis observed in our study compared to the absence of fibrosis in the acute setting of an earlier study [58]. Interestingly, our results showed that fibrosis levels decreased at 7 days compared to 3 day time point (Fig. 7A and B). These changes are also likely due to proteolytic actions of MMPs on provisional reparative fibrosis in the acute phase of Dox treatment, which may subsequently switch to a reactive phase of fibrosis in the long run under the influence of sustained ROS/RNS actions and associated secondary pathways such as inflammation and neurohumoral signalling events. Indeed, significance of such secondary events in reactive fibrosis is underscored by a relatively larger spread of Iso induced fibrotic lesions compared to that of Dox induced lesions at 7 day time points (Fig. 6E).

In this study we showed that levels of detergent soluble α-tubulin monomeric protein were significantly lower in Dox treated wild type heart lysates compared to those in control group at 3 day time point and these levels were restored back to control values at 7 day time point. These findings are consistent with a previous report which documented a similar decrease and restoration of α-tubulin levels in a rat model of Dox induced cardiotoxicity [36]. Although it was initially proposed that oxidative stress caused by Dox may be responsible for degradation of α-tubulin [36] or damage to microtubule system [37], more recent studies using various cancer cell lines have uncovered a direct link between p53 and microtubular network. Functional microtubules (polymers of α- and β- tubulins) and dynein were shown to participate in the nuclear transport of p53 after Dox treatment [63]. Upon entering the nucleus, p53 was shown to repress transcription of a microtubule associated protein 4 (MAP4) which is essential for stabilization of microtubule structures in the cytosol [64]. Consequently, downregulation of MAP4 protein was shown to increase monomeric pool of tubulins with a shorter half-life [65], which were long known to exert a negative feedback control on transcriptional rate of tubulin genes leading to decreased protein synthesis [66]. While our study has not examined ratios of polymerized vs. monomeric microtubule proteins, it is possible that Dox induced decrease in α-tubulin monomers may result from similar interactions between p53 and microtubule network in cardiomyocytes and vascular cells. Certainly MAP4 plays a critical role in stabilization of microtubules during pressure overload cardiac hypertrophy and associated contractile dysfunction [67]. Overexpression of MAP4 in adult feline cardiomyocytes was shown to increase the density of microtubule network [68]. In this context, it is of interest to note that α-tubulin levels also decreased in Dox treated p53 CKO hearts at 3 day time point and restored back to control values at 7 day time point. While this result may suggest a role for p53 independent pathways in regulation of microtubule stability, it does not rule out similar interactions between p53 and microtubule network in vascular cells. Given the well established role of cytoskeletal networks in regulation of cardiac contractility [69], changes in α-tubulin levels following Dox treatment may explain in part cardiac functional improvements observed in earlier studies [21], [23]. Further studies are required to understand mechanisms involved in Dox induced regulation of microtubule network and its role in cardiotoxicity.

Collectively, our results suggest that selective loss of p53 in cardiomyocyte compartment is not adequate to prevent excessive free radical generation, myocardial apoptosis, interstitial and perivascular fibrosis as well as microtubule changes following Dox treatment. Due to sustained myocardial fibrosis in p53 CKO hearts, we conclude that there are other p53 independent apoptotic pathways leading to cardiomyocyte apoptosis. Our data from p53 CKO cardiomyocytes suggests that excessive reactive oxygen/nitrosactive stress may directly trigger p53 independent cell death pathways in Dox induced cardiotoxicity. Further studies are required to identify the key components of p53-independent cell death pathways responsible for Dox induced cardiac fibrosis. Our findings also underscore the importance of vascular lesions in Dox induced cardiotoxicity and raise a cautionary note for future strategies involving p53 inhibitors for prevention of cardiac events in patients undergoing Dox therapy.
